This article has been retracted.

# Comprehensive Diagnostic Medical System Based on Notch1 Signaling Pathway to Inhibit the Growth of Small-Cell Lung Carcinoma

**DOI:** 10.1155/2022/2311471

**Published:** 2022-05-19

**Authors:** Xiaoli Zhang, Ziying Yu

**Affiliations:** ^1^Department of Pathology, The First Affiliated Hospital of University of South China, Hengyang 421001, Hunan, China; ^2^Department of Emergency, The First Affiliated Hospital of University of South China, Hengyang 421001, Hunan, China

## Abstract

With the gradual application of big data and other technologies to the medical field, more and more people tend to get online medical services. This article mainly studies the comprehensive diagnostic medical system based on Notch1 signaling pathway to inhibit the growth of small-cell lung carcinoma. In the experiment, we used the rapid thawing method to recover the cells and took the logarithmic growth phase cells for cell passage. We calculated the cell concentration and diluted the cells according to the experimental requirements. According to the standard curve, the corresponding sample protein concentration was calculated; at the same time, the Trizol method was used to extract the total RNA, the NanoDrop8000 spectrophotometer was used to determine the RNA concentration, and the RNA quality was detected by agarose gel electrophoresis. We used immunohistochemical staining to complete the staining of lung cancer cells. Finally, black box testing was used to test the functional modules of the system. Experimental data show that the accuracy rate of data obtained by the system reaches 98%, which greatly facilitates doctors and patients. The results show that the system has good ease of use and reliability and improves the diagnosis and treatment of hospital patients.

## 1. Introduction

In recent decades, while people's material living standards have improved, the incidence of many diseases has been increasing, including lung cancer. The Notch signaling pathway is more and more relevant to tumors, and it has become a hot spot in the field of tumor research. An important research topic of medical information science is to study medical diagnosis systems with intelligent diagnosis functions.

The role of Notch pathway in tumors can be used as either an oncogene or a tumor suppressor gene, which depends on the environment of tumor cells and its crosstalk with other signal pathways. It also facilitates distance education of medical staff to patients and improves the learning of new technology and business by the hospital's basic staff.

Notch1 is an important tumor suppressor gene. Jing et al. found that miR-140-5p was significantly downregulated in HSCC tissues and correlated with tumor classification and lymph node metastasis. The restoration of miR-140-5p inhibits the migration and invasion of FaDu cells and reduces the protein expression level of ADAM10. The factors considered in their research are not comprehensive [1]. Sui et al. believe that the pathway induced by Notch1 is related to cell growth, apoptosis, motility, and invasion in many cancers. They used an in vitro assay to detect the expression of Notch1 and NICD1 in hepatocellular carcinoma (HCC) tissues. Then, they used Notch1 siRNA or plasmids to explore cell biology and signaling pathways. There are certain flaws in their research [2]. Wu et al. studied the role of AITC in upregulating the expression of MRP1 and its relationship with the activation of the Notch1 signaling pathway by combining in vivo and in vitro experiments. They used Notch1 signaling pathway inhibitor DAPT to treat human bronchial epithelial cells to verify the effect of Notch1 on AITC-induced MRP1 expression. Their research lacks necessary experimental data [3]. Shi et al. believe that MicroRNA (miRNA) has become a new type of regulator in various pathological processes including ischemic stroke. However, the exact role of miRNA in ischemic stroke remains unknown. They investigated the role of miR-137 in regulating the effects of oxygen glucose deprivation and reoxygenation (OGD/R) on neuronal ischemia/reperfusion injury in a global cerebral ischemia model. Their research lacks innovation [4, 5].

This article establishes a quantitative medical knowledge base. Then, through the same method, we identify the user's symptoms, age, gender, and disease in the medical question and answer data, thereby establishing a quantitative relationship between disease and symptoms, age, and gender. Through the analysis and mining of data, the needs of the corresponding hospital patients can be further accurately analyzed, and appropriate and relevant supporting medical resources can be provided for some key medical institutions.

## 2. Notch1 Signaling Pathway and Small-Cell Lung Carcinoma

### 2.1. Notch1 Signaling Pathway

Notch protein is a transmembrane protein, which is composed of heterodimers generated by gene coding and plays a key role in cell proliferation. The basic unit is the extracellular domain, including the transmembrane domain, cysteine, and epidermal growth factor. In general, the transmembrane region combines with the heterodimer domain to form a noncovalent bond structure, which promotes the communication between the extracellular region and the thrombotic cell and plays a key role in activating Notch [6].

In some vertebrate Notch ligands, the C-terminus of the intracellular region contains a PDZL region, which can promote the adhesion of intercellular adhesion points and inhibit cell movement. It activates the Notch pathway by binding to the receptor, prompting the Notch receptor to release the intracellular region and enter the nucleus to play a role. And Hes1 is one of the important effector genes downstream of the Notch pathway, and its expression in malignant tumor cells can also change accordingly [7].

### 2.2. Small-Cell Lung Cancer

The intrinsic mechanisms of drug resistance include the change of drug transporter expression, activation promoting survival, anti-apoptotic pathway, and nonintrinsic influence of microenvironment of tumor. Obviously, tumors are heterogeneous cell populations with different genetic, epigenetic, and phenotypic characteristics. Different responses to treatment led to the emergence of resistant clones. Tumor heterogeneity is manifested in the ability of tumor cell subsets to drive cells and tumor initiation, high self-renewal, and multilineage differentiation. CSCs are associated with chemoresistance and radiotherapy resistance of NSCLC [8, 9].

Poorly differentiated squamous cell carcinoma is the least differentiated in squamous cell lung carcinoma. It is not only similar to small cell lung cancer in general but also more common in central type, and it is difficult to distinguish from small cell lung cancer under a microscope. The pathogenesis of the activation of the KRAS signaling pathway related to smoking and the activation of the EFGR signaling pathway related to nonsmoking are both found in lung adenocarcinoma. Squamous cell carcinoma is mostly located in the center, tends to spread along the airway and invade regional lymph nodes, and is prone to local recurrence. The basic principle of radiotherapy is segmented radiotherapy [10]. Reducing the dose per split will increase the tissue tolerance to radiation, and increasing the dose will cause serious late complications. In addition, the main reason for the low five-year survival rate of NSCLC patients is local recurrence or distant metastasis. At first, the mechanism of paclitaxel as a radiosensitizer was because it blocked the G2/M phase, but as follow-up research progressed, researchers found that its involvement in the radiation response was because it increased the reoxidation process of tumor cells. Reducing the oxygen consumption rate can block the respiration of tumor cells, thereby effectively reducing the number of tumor cells [11].

The treatment of NSCLC needs to integrate the diagnosis and treatment of various departments, including accurate diagnosis of imaging, pathology, inspection, and other departments, as well as comprehensive treatments such as surgery, radiation therapy, chemotherapy, targeted therapy, and immunotherapy, and the treatment of NSCLC is gradually moving towards personality. Radiotherapy is one of the most important treatments for NSCLC, participating in nearly 70% of NSCLC treatments. With the progress of radiophysics and radiobiology, radiotherapy has made great progress in the treatment of NSCLC. For early-stage patients, hyperfraction stereotactic radiotherapy can even achieve the same curative effect as surgery [12].

### 2.3. Comprehensive Diagnostic Medical System

The transmission distance between ZigBee network nodes is determined by the response speed of the received information and the transmission power, namely:

(1) $$\begin{array}{c} R=\frac{\lambda }{4\pi }\sqrt{\frac{P_{\text{tx}}}{P_{\text{rx}}}}, \end{array}$$

where *R* represents the coverage and *λ* represents the wavelength in the air medium.

Assuming that the node where the *k*-th ant is currently located is *i*, the probability of moving from this node to node *j* is

(2) $$\begin{array}{c} Pij=\left\{\begin{array}{c} \frac{\tau {\left(i,j\right)}^{\alpha }\cdot \eta {\left(i,j\right)}^{\beta }}{\sum_{u\in N_{k}^{i}}\tau {\left(i,u\right)}^{\alpha }\cdot \eta {\left(i,u\right)}^{\beta }},\\ 0, \end{array}\right. \end{array}$$

where *η*(*i*, *j*) is the heuristic information on the arc length (*i*, *j*).

The total change of pheromone on any arc (*i*, *j*) is

(3) $$\begin{array}{c} \Delta \tau \left(i,j\right)=\sum_{k=1}^{m}\Delta \tau_{ij}^{k}. \end{array}$$

First, the sum of the delays of each node *T* is shown in the following formula:

(4) $$\begin{array}{c} T=\sum_{i=0}^{N}T_{i},\\ E=\frac{1}{t}\times \sqrt{E_{0}}\times \alpha , \end{array}$$

where *N* is the number of transit hops in the route.

The remaining energy function, the number of hops, and the delay function constitute the pheromone increment function. Its expression is as follows:

(5) $$\begin{array}{c} \Delta \varphi_{n,d}=\frac{1}{\omega_{1}T+\omega_{2}N+\omega_{3}E^{-1}},\\ \varphi_{c,d}^{i+1}=\left(1-\lambda \right)\varphi_{c,d}^{i}+\Delta \varphi_{c,d}^{i},\\ P_{c,d}=\frac{{\left(\varphi_{c,d}^{i}\right)}^{\beta }}{\sum_{i\in M}{\left(\varphi_{c,d}^{i}\right)}^{\beta }}. \end{array}$$

The 5/3 filter is used in the system implementation, and the expression is as follows:

(6) $$\begin{array}{c} \chi \left(2n\right)=L\left(n\right)-\frac{H\left(n-1\right)+H\left(n\right)}{4},\\ \chi \left(2n+1\right)=\frac{L\left(n\right)+L\left(n+1\right)}{2}+\frac{-H\left(n-1\right)+6H\left(n\right)-H\left(n-1\right)}{8}. \end{array}$$

The spatial transformation of an image is a function that establishes the mapping relationship between an image and all points in the deformed image, namely:

(7) $$\begin{array}{c} \left[x,y\right]=\left[X\left(u,v\right),Y\left(u,v\right)\right],\\ \left[u,v\right]=\left[U\left(x,y\right),V\left(x,y\right)\right], \end{array}$$

where [*x*, *y*] represents the coordinates of the pixels in the input image and [*u*, *v*] represents the coordinates of the pixels in the output image.

Most of the spatial transformation can be represented by a 3^∗^3 transformation matrix:

(8) $$\begin{array}{c} \left[x^{\prime },y^{\prime },w^{\prime }\right]=\left[u,v,w\right]T. \end{array}$$

Among them,

(9) $$\begin{array}{c} T=\left[\begin{array}{ccc} a_{11} & a_{12} & a_{13}\\ a_{21} & a_{22} & a_{23}\\ a_{31} & a_{32} & a_{33} \end{array}\right],\\ \left\{\begin{array}{c} x=\frac{x^{\prime }}{w^{\prime }},\\ y=\frac{y^{\prime }}{w^{\prime }}, \end{array}\right. \end{array}$$

where *T* is called the transformation matrix and *x*, *y*, and *u*, v are the coordinates before and after the transformation.

The overall architecture of the medical system is shown in Figure 1. It can be seen from the figure that the visualized interactive medical system realizes the visualization of medical image processing [13].

The business logic of a hospital website or the back-end management system of a medical institution can be divided into two parts:

1. From the perspective of system functions, some common functions can be added to the framework, which also includes website business logic functions and hospital management system business logic functions [14].
2. From the perspective of the department setting of medical institutions, with department as the unit, corresponding functional modules are set up, but whether it is the department module or the specific function subsystem, each part of the system is relatively independent, which allows developers to flexibly combine through configuration [15, 16].

The telemedicine diagnosis system is shown in Figure 2. Medical conference and remote consultation system is essential for digital hospitals. Many hospitals have installed network conference system, but these systems do not have professional medical consultation process management, docking function with medical equipment, and synchronous recording function of video and audio medical information. Based on the “unified communication” of international standard, a consultation conference system with complete medical professional functions is designed for professional medical consultation. It can be used not only as an auxiliary system for surgery and treatment in the hospital but also as a live broadcast system for large-scale medical academic conferences.

The system structure model is shown in Figure 3. In the conference management module, its main function is to call the functions of the data network layer to complete the conference management, maintain the information of the conference node, and invite the node to open the session. In the conference data transmission module, its main function is to complete the message transmission between conference participants through the services provided by the data distribution network. The data transmission function of service layer is suitable for complex network transmission environment. As a clinical application information system that provides comprehensive clinical information services to clinical medical staff, the design and function realization of medical diagnosis system need to fully consider and meet the clinical work and related extension work around the clinical work and need to meet the needs of medical, nursing, and technical personnel, patient-centered, providing timely clinical information for users in clinical medical services. It needs to be consistent with the habit and logic of clinical work, and it needs to meet the needs of providing auxiliary decision making based on the logical guidance of clinical affairs and the advantages of intelligent computing technology.

The architecture of wireless medical video monitoring system is shown in Figure 4. Through the framework of broadband wireless local area network (WiFi), 802.11 as the wireless connection protocol, it supports the interconnection protocol DLNA, IGRS, and even UPnP, supports the use of video monitoring equipment supporting wireless broadband routing, sets up wireless cameras in the designated monitoring points of the ward, and transmits images to the monitoring screen of the nurse station through the wireless device, so as to facilitate doctors and nurses to communicate with patients. It can also observe the actual situation of patients in the ward for real-time monitoring. At the same time, the wireless secure storage system (WSS) can automatically receive the images transmitted by wireless, so that the doctors on duty and attending doctors can know the patient's condition and status off-site and even obtain the needed real-time images and retrieve and query the historical images through the Internet.

The architecture of medical cold chain and environmental monitoring management platform is shown in Figure 5. As a professional medical aid unit, 80% of the medical staff in hospitals are engaged in medical activities, and they have no time to take care of extra matters. Due to the large number of hospital medical equipment and information systems and limited management personnel, they are often in a state of no supervision, such as ultra-low temperature refrigerators, liquid nitrogen tanks, and other valuable equipment and facilities and areas. Even if the monitoring platform is introduced for real-time monitoring, there is no special person to track and supervise the whole process. In addition, the monitoring platform also needs professional operation and maintenance, and some medical equipment and facilities monitored also need to carry out metrological verification every year, and new equipment procurement also needs to carry out model selection, incoming inspection, and initial setting. These contents are far beyond the scope of medical institutions.

## 3. Notch1 Signaling Pathway Inhibits the Growth of Small-Cell Lung Cancer

### 3.1. Subjects

134 cases of primary lung cancer were selected as archived wax blocks, including 36 cases of small-cell lung carcinoma and 98 cases of squamous cell carcinoma. In addition, about 10 slices of 10 *μ*m thickness were cut for flow cytometry.

### 3.2. Experimental Instruments and Reagents

The main instruments used in the experiment are upright ordinary optical microscope, manual tissue chip instrument, precast wax block, electric heating incubator, anti-dropping glass slide, cover glass, etc.

The main reagents used in the experiment are Notch1 antibody, SP-9000 immunohistochemical detection kit, DAB color reagent kit, PBS buffer, citrate buffer, etc [17].

### 3.3. Cell Culture

1. Cell resuscitation: cells were resuscitated by the rapid melting method. Take out H1299 cell and A549 cell cryopreservation tube, respectively, from liquid nitrogen container, put them into 37°C water bath quickly, make the cells melt completely in 1-2 minutes, sterilize the tube mouth with 75% alcohol, absorb the melted cell suspension, and transfer it into 10 ml centrifuge tube. Then, 10 times the volume of the mixture was centrifuged at 1000 rpm for 5 minutes at room temperature to remove DMSO from the cryopreservation solution [18].
2. Cell passage: take the logarithmic growth phase cells, discard the supernatant, add 1 ml 0.25% trypsin into the culture bottle to digest the cells, put them in the incubator, set the temperature at 37°C, digest for 1 min, and observe closely under the inverted microscope until the peripheral contour of the cells shrinks and becomes round; the DMEM medium is added immediately to terminate the digestion reaction [19].
3. Cell count: after the cells are digested with trypsin, when the cells do not fall obviously, discard the trypsin, dilute the cells with a certain amount of culture medium, and fully blow them out with a pipette. After estimating that the cells are single, take 100 *μ*L cell suspension in the EP tube and mix them gently. After blowing the gun head gently, draw 20 *μ*L cell suspension from it into a specific cell counting plate, put it into the instrument, count the cells, count three fields of vision for each sample, and take the average value. The cell concentration was calculated and the cells were diluted according to the experimental requirements [20, 21].

### 3.4. Western Blot

The BCA method was used to determine the protein concentration. Preparation of protein standard solution: 5 mg/ml protein standard solution was diluted by multiple ratio, and water bath was conducted at 37°C for 30 min. According to the standard curve, the corresponding protein concentration was calculated. When the concentrated gel polymerizes, pull out the Teflon comb, take 20∼100 *μ*g protein sample, load the sample according to the predetermined sequence, and add 1 × SDS sample loading buffer into the blank hole to make up the volume [22, 23].

### 3.5. Trizol Method to Extract Total RNA

The cells were centrifuged at room temperature at 1500 rpm for 5 min. The supernatant medium was discarded and the cells were collected. The cells were resuspended with 1 ml of precooled Trizol, and the cells were left for 5 min at room temperature. Add 200 *μ*l chloroform, shake violently for about 15 sec, and let stand for 5 min. The supernatant was centrifuged at 4°C for 15 min at 12,000 rpm. The NanoDrop8000 spectrophotometer was used to determine RNA concentration. Agarose gel electrophoresis was used to detect the quality of RNA, and it is stored at −80°C and kept standby [24].

### 3.6. Cell Staining

The liposome transfection method is used to co-transfect the reporter gene plasmid and the gene expression plasmid or its control plasmid into the cells. Immunohistochemical staining was used to complete the staining of lung cancer cells. Paraffin specimens 4 *μ*m thick sections are routinely deparaffinized to water. Hot antigen retrieval requires more than 20 minutes at a temperature of 95°C, and then stir at room temperature for at least 30 minutes. Hematoxylin lightly stains the nucleus for 5–10 seconds, conventionally dehydrated, transparent, and mounted [25].

### 3.7. Statistical Analysis

Statistical analysis was carried out using SPSS18.0 software. After the homogeneity of variance test, the one-way ANOVA and SNK-q test were used for analysis. The survival curve was analyzed by long-rank test, and the weight change was analyzed by the area under the curve. For the relationship between Notch1 expression and clinicopathological characteristics in small-cell lung cancer, we used *t*-test to compare the two sets of data. *P* < 0.05 is considered statistically significant [26].

### 3.8. System Test

#### 3.8.1. Simulation Model Parameters

In the cell model process, we use the urban micro model to simulate three eNodeB nodes, and five UEs per node. Moreover, the UE moves radially from the center to the four sides at a speed of 15 km/h [27]. The simulation model parameters of the system are shown in Table 1.

#### 3.8.2. System Test

In this paper, we use the function test to test the system. The tested program is like a black box that cannot be seen. The tester does not know or need to know the internal structure, source code, and programming language of the program in advance. He only needs to know what functions the program wants to realize and how to operate the program input and output. The tester tests the interface and function of the program by inputting data at the program interface to see whether the output data are correct and whether they meet the requirements of software design. The connection verification of the server in different platforms is successful, the network communication is smooth, there is no packet loss phenomenon, and the breakpoint connection can be realized. Remote system control of the client can realize remote login, obtain permissions, and maintain and manage the server [28–30].

## 4. System Test Results

### 4.1. Comprehensive Diagnostic Medical System Test Results

In order to verify the effectiveness of the algorithm, the NS2 simulation platform is used to design simulation rules, and the network is carried out in the range of 500^∗^500. The maximum number of nodes in the network is 60. The maximum transmission distance of the node in the space is 50 meters, the rate is 250 kbps, the channel delay is set to 0.3 s, and the data packet length is set to 128 bit. Before starting the experiment, the initial value of energy given to the whole network is 10000 units, and each node consumes 1 and 2 energy units when receiving and sending a packet. The time of each experiment is 200 seconds, and the average value of 30 experiments is taken. The comparison of network energy consumption is shown in Figure 6. The ACO-AODV algorithm routing greatly reduces the overall energy consumption of the network, which is achieved by avoiding the connection of low energy nodes for the number of hops and delays in the process of exploring the path. But after particle swarm algorithm and genetic algorithm are run, the effect of optimization of energy consumption is not significant.

When a patient has an emergency, the monitoring center needs to be able to detect and notify the doctor and patient in time. This requires the system to transmit the patient's physiological parameters in real time and process the response feedback in real time. Usually, there is a delay in the transmission and processing of physiological parameters, but the delay must be controlled within a certain range. The transmission processing delay time required by this system must be less than 3 seconds. The system test results are shown in Table 2. It can be known from the test results that the system fully implements a wireless sensor device network remote medical supervision and nursing system. The result shows that the accuracy rate of the data obtained by the system reaches 98%, which greatly facilitates doctors and patients.

When the distance between the patient and the host computer is about 5 meters and in an indoor environment, different timers are set to test at different data collection frequencies. The terminal node sends physiological data to the coordinator node, summarizes whether there is storage overflow according to the test results, and calculates the packet loss rate and makes statistics as shown in the following table. The data transmission rate verification results are shown in Table 3 and Figure 7. The results show that the packet loss rate of data transmission is positively correlated with the sending frequency of data packets, that is, the higher the sending frequency of data packets, the higher the packet loss rate because when the collection speed is too fast, storage overflow is prone to occur, and the data are too late to be sent. The new data to be stored came again, causing the original data to be overwritten.

### 4.2. Mechanism of Notch1 Signaling Pathway on Small-Cell Lung Carcinoma

To verify the expression of Notch1 in lung tissue, we used immunohistochemistry to detect the expression of Notch1. The results of immunohistochemistry are shown in Figure 8. There was a small amount of Notch1 protein expression in the control group, and a large amount of PDGFR*β* protein expression in lung tissues could be seen in the model group.

The effects of Cur combined with VCR on mRNA expression of Notch1, Jagged1, and Hes1 in Eca-109/VCR cells are shown in Table 4 and Figure 9. The results showed that the mRNA expression levels of Notch1, Jagged1, and Hes1 in the Cur group were 0.917 ± 0.033, 0.817 ± 0.069, and 0.860 ± 0.055, respectively, and those of Notch1, Jagged1, and Hes1 in the VCR group were 0.874 ± 0.059, 0.798 ± 0.055, and 0.696 ± 0.038, respectively. The mRNA expression levels of Notch1, Jagged1, and Hes1 in the Cur + VCR group were 0.506 ± 0.054, 0.349 ± 0.045, and 0.529 ± 0.045, respectively. Compared with the control group, the mRNA expression levels of Notch1, Jagged1, and Hes1 in the Cur group, VCR group, and Cur + VCR group were decreased (*P* < 0.05); compared with the Cur group and VCR group, the mRNA expression levels of Notch1, Jagged1, and Hes1 in Cur + VCR group were significantly decreased (*P* < 0.01).

After 5-FU treatment, the apoptosis of HCC cells was detected by the AnnexinV-APC/PI double labeling method. The results showed that compared with the control group, the percentage of apoptotic cells in the knockdown of Notch1 expression was significantly increased, and the number of apoptotic cells decreased again after the expression of Notch1 was restored. Under normal physiological conditions, epithelial-mesenchymal transition (EMT) is very important for mammalian embryonic development. After adulthood, its activity stops. However, during tumor growth, this process is activated again. The activated EMT changes the morphology of tumor cells and realizes the migration ability of tumor cells through the loss of epithelial cell polarity. At the same time, the expression of E-cadherin, N-cadherin, and vimentin changes. The invasion and metastasis of tumor cells were enhanced. Notch signaling pathway is an evolutionarily highly conserved signaling pathway, which participates in various processes of cell activity, including cell life span, tissue morphology, and cell differentiation, proliferation, and death.

### 4.3. Inhibition of Notch1 Signaling Pathway

RT-PCR was used to detect the expression of Egf17, Notch1, E-cadherin, protein, and vimentin mRNA in 40 cases of NSCLC and 20 cases of normal lung tissue adjacent to cancer. The results are shown in Table 5. The results showed that the expression levels of Egf17, Notch1, and vimentin mRNA were lower in normal lung tissues and higher in NSCLC tissues; the expression levels of E-cadherin mRNA in NSCLC tissues were 3.403 ± 0.181 and 5.748 ± 0.72 in normal lung tissues. The results of immunohistochemistry and RT-PCR showed that Egf17, Notch1, E-cadherin, and vimentin protein expressions were consistent in NSCLC tissues and adjacent normal lung tissues, that is, the positive expression rate and mRNA expression of Egf17, Notch1, and vimentin in NSCLC tissues were higher than those in adjacent normal lung tissues. The positive expression rate and mRNA level of E-cadherin protein and mRNA in NSCLC tissues were lower than those in adjacent normal lung tissues (*P* < 0.05).

In order to determine the best concentration of Notch1 specific inhibitor LY3039478, we set three inhibitor concentration gradients of 6 mg/kg, 8 mg/kg, and 10 mg/kg and used western blot to detect the expression of Notch1 to determine the best inhibitor concentration. The result is shown in Figure 10. Compared with the ICH group, the overexpression of HIF-2*α* significantly increased the expression level of CD31. However, Notch1 inhibitors effectively inhibited the upregulation of CD31 by HIF-2*α*. At the same time, compared with the ICH group, Notch1 inhibitors can effectively reduce the expression of CD31.

For lung cancer EC-97006 cells, preventing the expression of Notch1 can prevent the emergence of EMT, and it can also weaken the characteristics of spread and invasion. When EC-97006 cells were transfected with siNotch1, the expression level of E-cadherin increased, and the expression level of vimentin decreased. Notch1 plays a key role in the process of EC-97006 cell proliferation and invasion. The expression of Notch1 is shown in Figure 11. The positive expression rate of Notch1 in the wild group was 26.34%, the positive expression rate in the mutant group was 39.29%, and the positive expression rate in the drug-resistant group was 47.39%. And EGFR is widely expressed in most hypopharyngeal carcinoma tumor tissues.

### 4.4. System Performance Comparison

This test uses 10 virtual users to test Struts framework at the same time. At the beginning, users are allowed to increase 2 users every 2 seconds. This operation is repeated. When the number of users reaches 10, the test process is run, and the test time is set to 2 minutes, that is, the time for 10 people to conduct transaction test at the same time is 2 minutes. When the number of users is reduced to 0, the test is stopped.  Table 6 and Figure 12 show the service response time of prescription submodule implemented by Struts framework. According to the above data, we can see all the data information related to this test. The shortest transaction response time is 8.04 seconds, the longest transaction response time is 8.138 seconds, and the average transaction response time is 8.07 seconds.

Firstly, in the initial stage, we use all the features to establish a random forest classification prediction model based on 10 times cross-validation. Then, the importance of each index is sorted, and the most appropriate number of features is selected to form the best prediction performance. In the second stage, various models are constructed by using adjustable parameters, which are adjusted on the basis of increasing the number of top features. The step size of ntree is adjusted from 500 to 2000, increasing by 100 per step; once ntree value is fixed, mtry increases from 2 to 15 by increasing 1 per step. In the final stage, based on the principle that the number of features is the least but the prediction performance is the same as the overall index, the final model consists of 17 features, and ntree and mtry are 1200 and 7, respectively. The feature selection process is helpful to select the most valuable information related to gastric cancer from the blood test indicators. At this time, the accuracy of Co-SVM algorithm is the best, which has reached 85.556%. Compared with the support vector machine algorithm commonly used in the auxiliary heart disease diagnosis system, the accuracy rate of neural network algorithm is improved by 1.6 percentage points; the classification accuracy of neural network algorithm is 77.78% and that of the decision tree algorithm is 80.37%. The Co-SVM algorithm proposed in this paper is superior to other classical algorithms in terms of the main accuracy.

## 5. Conclusions

Notch1 signaling pathway is involved in the occurrence and development of PF. Blocking this pathway can reduce the production of myofibroblasts, inhibit epithelial-mesenchymal transition (EMT), and delay the development of PF. Notch1 signaling pathway can not only regulate cell-to-cell connections, signal transduction in the cytoplasm, and gene transcription in the nucleus but also affect cell activities. The apoptosis rate and proliferation activity of small-cell lung carcinoma are higher than those of squamous cell carcinoma and higher than those of normal lung tissue. In squamous cell carcinoma, the apoptotic rate and proliferation activity increase with the grade.

The telemedicine system in this paper is based on C/S architecture. The system adaptability of C/S architecture is stronger, and it is easier to deal with many professional problems such as medical image display, rapid file transmission, information sharing, electronic settlement, and medical activities, so that users can better complete telemedicine activities and improve work efficiency. At the same time, the related functions of remote consultation business system are realized, and the principle of database construction is briefly described.

In the implementation, we store all kinds of media information in the background relational database. For large capacity video and audio information, how to store more effectively in the database is a problem worthy of discussion. Using the media information stored in the database to support streaming media is also a challenging topic. Using JMF to build push data source can provide convenience for the transmission of video and audio stream, and it will provide better help for the client to process multimedia information better. The integration of this system and telemedicine system is conducive to the sharing of patient information. Experts can make full use of it and PACS data resources and can effectively maintain the authenticity of video and image data.

## Figures and Tables

**Figure 1:** The overall architecture of the medical system.

**Figure 2:** Telemedicine diagnosis system.

**Figure 3:** System structure model.

**Figure 4:** Architecture of wireless medical video monitoring system.

**Figure 5:** Architecture of medical cold chain and environmental monitoring management platform.

**Figure 6:** Comparison of network energy consumption.

**Figure 7:** Data transfer rate verification result.

**Figure 8:** Immunohistochemistry results.

**Figure 9:** The combined effect of Cur and VCR on the mRNA expression of Notch1, Jagged1, and Hes1.

**Figure 10:** Expression results of Notch1.

**Figure 11:** Expression of Notch1.

**Figure 12:** Business response time of the prescription submodule implemented by the Struts framework.

**Table 1:** Simulation model parameters of the system.

Parameter	Urban macro community
Road loss model scenario	Urban_micro
Base station spacing	500 m
Duplex mode	TDD
Channel model	PedB
Carrier frequency	2 GHz
Bandwidth	20 MHz
Subcarrier width	180 kHz
Frequency reuse factor	1
Amount of users	5

**Table 2:** System test results.

Project	1	2	3	4	5	6	7	8	9
Packet loss rate	8.5%	5.5%	4.9%	7.7%	8.1%	3.2%	2.2%	5.1%	2.6%
Accuracy	91%	93%	89%	89%	95%	98%	96%	94%	97%

**Table 3:** Data transmission rate verification results.

Frequency	35	37	66	63	36	35	31	36	59	57
Packet loss rate	3.79%	2.64%	4.31%	3.12%	3.94%	4.45%	3.56%	5.04%	5.49%	4.75%

**Table 4:** The combined effect of Cur and VCR on the mRNA expression of Notch1, Jagged1, and Hes1.

Group	Notch1	Jagged1	Hes1
Control	1.000	1.000	1.000
Cur	0.917 ± 0.033	0.817 ± 0.069	0.860 ± 0.055
VCR	0.874 ± 0.059	0.798 ± 0.055	0.696 ± 0.038
Cur + VCR	0.506 ± 0.054	0.349 ± 0.045	0.529 ± 0.045

**Table 5:** Expression of Egf17, Notch1, E-cadherin, and vimentin mRNA in lung tissues of each group.

Organization type	Egf17 mRNA	Notch1 mRNA	E-cadherin mRNA	Vimentin mRNA
Normal lung tissue	3.417 ± 0.76	4.217 ± 1.27	5.748 ± 0.72	2.243 ± 0.73
Lung cancer tissue	6.88 ± 0.62	6.791 ± 1.52	3.403 ± 0.181	5.812 ± 0.36

**Table 6:** Business response time of prescribing submodule implemented by Struts framework.

Times	Shortest response time	Longest response time	Average response time	Simulation consideration time
1	8.04	8.138	8.07	8
2	8.025	8.108	8.041	8
3	8.024	8.178	8.052	8
4	8.027	8.714	8.092	8
5	8.03	8.155	8.076	8
6	8.032	8.111	8.063	8
7	8.027	8.175	8.058	8
8	8.028	8.274	8.074	8

## Data Availability

The data that support the findings of this study are available from the corresponding author upon reasonable request.
